The article "MiR-212-3p promotes proliferation and migration of trophoblast in fetal growth restriction by targeting placental growth factor" was published in 2021. Journal: Bioengineered.

# MiR-212-3p promotes proliferation and migration of trophoblast in fetal growth restriction by targeting placental growth factor

**DOI:** 10.1080/21655979.2021.1967069

**Published:** 2021-09-02

**Authors:** Limin Yu, Yan Sun, Zanjun Chu

**Affiliations:** Department of Gynecology and Obstetrics, Tianjin Medical University General Hospital, Tianjin, China; Tianjin Key Layboratory of Female Reproductive Health and Eugenics, Tianjin, China

**Keywords:** Fetal growth restriction, miR-212-3p, PGF, PI3K/AKT signaling pathway, biomarkers

## Abstract

The purpose of this study was to evaluate the function and possible mechanism of miR-212-3p in fetal growth restriction (FGR) and to demonstrate the relationship between miR-212-3p and placental growth factor (PGF). First, we used qRT-PCR to detect the expression of miR-212-3p and PGF in placental tissues of normal delivery (HC group) and FGR, as well as in human trophoblast cell HTR-8/Svneo. The results revealed that miR-212-3p expression was significantly upregulated and PGF was significantly downregulated in placental tissue in the FGR group compared with the HC group. In addition, interference with miR-212-3p expression increased the proliferation, invasion, and migration of HTR-8/SVneo cells and decreased apoptosis of cells. Meanwhile, Western blot results showed that miR-212-3p expression downregulation promoted the phosphorylated protein expression of Phosphoinositide 3-kinase (PI3K) and protein kinase B (AKT), which in turn activated the PI3K/AKT signaling pathway. And the results of dual luciferase reporter further showed that miR-212-3p could target PGF, and the expression of both was negatively correlated in FGR group tissues. In addition, downregulation of miR-212-3p expression reversed the inhibitory effect of PGF downregulation on HTR-8/SVneo cells. In conclusion, miR-212-3p can target and inhibit the PGF expression and regulate the PI3K/AKT signaling pathway to regulate trophoblast cell invasion, migration, proliferation and cell apoptosis. This provides a potential biomarker for the development of FGR.

## 1. Introduction

Uteroplacental disorders such as placental hypoxia or hypoxia result in abnormal trophoblast function, which in turn triggers many complications, such as preeclampsia and fetal growth restriction (FGR) [1,2]. According to the definition of the Royal College of Obstetricians and Gynecologists and the American College of Obstetricians and Gynecologists, FGR, known as intrauterine growth retardation, is described as that the fetus is unable to grow normally in the uterus for various adverse reasons, shown by fetal weight and abdominal circumference below 10% of the normal standard of its gestational age [3–6]. So far, FGR remains a global issue and the main reason for the morbidity and mortality of the perinatal fetus and neonate. Epidemiological survey statistics have found that the mortality rate caused by FGR is up to 30% [7], therefore, screening for FGR is essential.

MicroRNAs (miRNAs), a type of endogenous non-coding molecule with 18–25 nucleotides, regulates a series of processes by specifically binding to the 3ʹ-UTR of mRNAs including apoptosis, gene expression, proliferation and cell differentiation [8]. So far, more than 700 miRNAs have been mined, and abnormal expression of some miRNAs has been found to lead to multiple complications during pregnancy and trigger a variety of pathologies, for example like FGR, preeclampsia, and gestational diabetes, and it is of great importance in predicting therapeutic strategies and targeted therapy [9–11]. Currently reported miRNAs associated with placental dysfunction are miR-424 [12], miR-18a-5p [13], miR-149 [14], miR-133a [15], and miR-98 [16]. For example, Zou et al. found that miR-424 could regulate the proliferation and invasion of trophoblast cell lines and mediate the expression of protein ERRγ and HSD17B1, which took part in the development of FGR [12]. Zhang et al. [13] found that H19 down-expressed inhibits trophoblast cell proliferation and invasion and is involved in the molecular mechanisms regulating FGR by targeting miR-18a-5p. Gao et al. [14] found that cell proliferation and invasion were inhibited by miR-149 through targeting inhibition of placental growth factor (PGF) expression. In addition, it has been shown that miR-212-3p has attended regulation of the development of osteosarcoma, glioblastoma, as well as gastric cancer, and is used as a molecular marker, so being as one of the important miRNA, miR-212-3p has a link with disease development [17–19]. In addition, Rodosthenous et al. [20] found that miR-212-3p was highly expressed in maternal serum with abnormal fetal growth. However, there is no literature report about the specific function and mechanism of miR-212-3p in FGR. In addition, we predicted PGF as one of the miR-212-3p target genes by bioinformatics in the previous stage. And PGF is now a key diagnostic marker for severe FGR or eclampsia [21]. Based on this, we speculate that miR-212-3p may be highly expressed in FGR and involved in FGR pathogenesis by regulating the expression of PGF. Therefore, the purpose of this article was to reveal the potential influence of miR-212-3p as well as PGF expression on invasion, apoptosis, and migration of the trophoblast cell line, and to assess their exact effect on FGR pathogenesis, which can support the theory of the great promoting influence of miR-212-3p on the FGR development, offering a theoretical reference for preventing and curing FGR.

## 2. Materials and methods

### 2.1. Placental tissue collection

Placental tissues with FGR and normal placental tissues that underwent delivery in our hospital from August 2017 to August 2019 were collected. The study was approved by the Medical Ethics Committee of Tianjin Medical University General Hospital (IRB2020-WZ-196), and all participants signed a written informed consent form.

### 2.2. Cell culture and transfection

We obtained HTR-8/SVneo cells from Shanghai Cell Research Institute (Shanghai, China). HTR-8/SVneo cells were cultured in DMEM high-glucose culture medium (Thermo Fisher Scientific, Waltham, USA) containing 1% penicillin/streptomycin (Gibco, Grand Island, USA) and 10% fetal bovine serum (FBS, Gibco, USA), and maintained in an incubator (Thermo Fisher Scientific, Waltham, USA) at 37 °C with 5% CO_2_.

HTR-8/SVneo cells transfection was performed using Lipofectamine 2000 (Invitrogen, CA, USA) following the instruction. MiR-212-3p inhibitor, NC inhibitor and PGF interference fragment PGF siRNA were synthesized by Guangzhou Ruibo Biotechnology Co., Ltd (Guangzhou, China).

### 2.3. Real-time quantitative fluorescence PCR (qRT-PCR)

A Total RNA extraction kit (Invitrogen, USA) was used to extract total RNA from tissues and cells. The RNA was converted into cDNA using by the instruction of reverse transcription kit (Takara, Japan). Followed by the instruction of the real-time PCR kit (Takara, Japan), the experiment was performed by using cDNA, and the reaction system was as followed: 95 °C for 1 minute; 35 cycles of 95 °C for 40 seconds, 58 °C for 40 seconds, and 72 °C for 45 seconds; and 72 °C for 10 minutes. With either the GAPDH or U6 selected as an internal reference, we used 2 ^−ΔΔCt^ method for data analysis. The primer sequence was shown in Table 1.

**Table 1.** Primer sequences of qRT-PCR

Gene Name	Primer Sequence (5ʹ-3ʹ)
PGF	F GTCTTCATTCCATCACTCTTCTTG
	R TCAGTGGT—GCTCCATACAGAAC
miR-212-3p	F GTCGTATCCAGTGCAGGGTCCGAG
	R TGGTTCGTGGGTAACAGTCTCCAGTC
U6	F CTCGCTTCGGCAGCACA
	R AACGCTTCACGAATTTGCGT
GAPDH	F TCAGTGGTGGACCTGACCTG
	R TGCTGTAGCCAAATTCGTT

### 2.4. MTT assay

Transfected HTR-8/SVneo cells were collected, and the cells were digested to 1 × 10^4^ cells/ml by trypsin and placed into a microplate with 96 wells. We transferred 20 μl MTT solution (5 mg/ml) to each well and cultured the plate for 4 h after incubation for 24, 48 and 72 h, respectively. After removing the supernatant, 150 μl DMSO was transferred to each well and mixed well for 5 min at room temperature. And then we used a microplate reader (Bio-Rad, USA) to measure the 490 nm absorbance value.

### 2.5. Flow cytometry

By using an AnnexinV-allophycocyanin (BD Pharmingen, SanJose, USA) apoptosis detection kit, apoptosis was detected. Cells were trypsinized and centrifuged, and the cells were washed twice using pre-cooled sterile PBS buffer. 1 × Binding Buffer was used to prepare cells of 1 × 10^6^ cells/ml. Operate in strict accordance with the instructions for use of the kit, add AnnexinV and nucleic acid dye into the cells, gently mix them, and place them in darkness at room temperature for 15 minutes; add 5 µl PI, and place them in darkness at room temperature for 15 minutes. They were subsequently tested on a FACScanflow cell flow system (BectonDickinson, SanDiego, CA, USA).

### 2.6. Transwell assay

500 μl of 10% FBS were transferred into the lower chamber of the transwell inserts (BD Biosciences, USA), 100 μl of diluted HTR-8/SVneo cells were transferred into the upper chamber, and then cultured it in an incubator which contains CO_2_ of 5% for 48 h at the temperature of 37 °C. The cells did not migrate during the time were wiped off from the layer of the upper part by a cotton swab, and then fixed with methanol, stained with crystal violet, observed and counted under a microscope. Ten fields were selected for observation, counting, and taking the mean value.

In the invasion assay, HTR-8/SVneo were transferred into the chamber of its upper chamber of the transwell coated by Matrigel (BD Biosciences, USA), and 10% FBS medium was added into its lower chamber. After culturing for 48 h, Matrigel glue and uninvaded cells were wiped off, fixed with methanol and stained. The counts were observed under a microscope.

### 2.7. Dual-luciferase reporter assay

When HTR-8/SVneo cells has reached the confluency of 80%-90%, the transfection would be performed. The constructed Dual-Luciferase Reporter Vectors of the mutant (PGF-MUT) and the wild-type (PGF-WT) were co-transfected with miR-212-3p mimics or NC mimics into HTR-8/SVneo cells, respectively, and cultured for 48 hours. After collecting the cells, we detected the luciferase activity by using a luminescence analyzer after the addition of luciferase substrate, and calculated the relative luciferase activity by using Renilla luciferase activity as an internal reference [22].

### 2.8. Western blot

Proteins were isolated from cells and placental tissues by utilizing the RIPA lysate (Sigma, USA), and the concentrations of protein was measured by a BCA protein assay kit (Beyotime, China). After SDS-PAGE separation, the proteins were blotted onto PVDF membranes. After blocking with 5% skimmed milk at oom temperature for 1 h, the membranes were incubated with primary antibodies PGF (Abcam, UK), Phosphoinositide 3-kinase (PI3K; #4249, Cell Signaling Technology, USA), p-PI3K (ab278545, Abcam, UK), β-actin (ab8226, Abcam, UK), protein kinase B (AKT; #4685, Cell Signaling Technology; USA) and p-AKT (#4060, Cell Signaling Technology, USA) at 4°C overnight. Till next day, the membranes were washed twice, secondary antibodies which were labeled by enzyme and diluted were added, and incubated at room temperature for 1 h. The color development was done by chemiluminescence, and the results analysis was performed by gel imaging system. β-actin was selected as an internal reference protein.

### 2.9. Statistical analysis

By making use of SPSS 22.0 software, two-sample mean T-test and one-way analysis of variance were performed. The results were displayed as the form of mean ± standard deviation (SD). It was believed to be significantly different when P < 0.05.

## 3. Results

### 3.1. MiR-212-3p was up-regulated in placentas tissues with FGR

First we wanted to determine the expression of miR-212-3p in FGR. The results of qRT-PCR showed that the miR-212-3p expression in placental tissues with FGR was notably increased by comparison with normal placental tissues in the HC group (Figure 1, p < 0.001). This result suggests that miR-212-3p is involved in the course of FGR.

**Figure 1.** qRT-PCR detection of miR-212-3p expression in placenta tissues of HC group and FGR group

### 3.2. Promotion of the invasion, migration and proliferation of HTR-8/SVneo and apoptosis inhibition by down-regulation expression of miR-212-3p

To determine the effect of miR-212-3p during FGR, loss-of-function experiments was accomplished by interfering with the miR-212-3p expressing in HTR-8/SVneo. RT-qPCR results indicated that comparing to NC group, miR-212-3p inhibitor significantly reduced miR-212-3p expression in HTR-8/SVneo cells (Figure 2(a)). MTT assay results showed that the cell proliferation rate of the miR-212-3p inhibitor group was notably higher by comparing to the NC inhibitor group (Figure 2(b)). Flow cytometry assay results showed that comparison with the NC inhibitor group, the cell apoptosis rate was significantly decreased in the miR-212-3p inhibitor group (Figure 2(c)). The results of transwell assay revealed that HTR-8/SVneo cells invasion and migration in the miR-212-3p inhibitor group were increased by comparing to the NC inhibitor group (Figure 2(d)). These results suggest that miR-212-3p down-expressed promotes trophoblast cell proliferation, migration and invasion, while inhibiting apoptosis.

**Figure 2.** Promotion of the invasion, migration and proliferation of HTR-8/SVneo and apoptosis inhibition by down-regulation expression of miR-212-3p

(a) Transfection efficiency of miR-212-3p in HTR-8/SVneo detected by qRT-PCR; (b) Cell proliferation detected by MTT assay; (c) Apoptosis detected by flow cytometry; (d) Cell invasion and migration detected by Transwell assay. **P < 0.01 and ***P < 0.001.

### 3.3. miR-212-3p downexpressed activats the PI3K/AKT signaling pathway

We used western blot to detected the key molecules expression of PI3K/AKT pathway (p-PI3K/PI3K and p-AKT/AKT). The results indicated that the p-AKT and p-PI3K expression were notably increased and the p-AKT/AKT along with p-PI3K/PI3K ratios was distinctly increased in the miR-212-3p inhibitor group when comparing to the NC inhibitor group (Figure 3). The above results revealed that down-regulation expression of miR-212-3p could increase the protein expression levels of p-PI3K and p-AKT in HTR-8/SVneo cells which in turn activated the PI3K/AKT signaling pathway.

**Figure 3.** Activation of the signaling pathway of PI3K/AKT by down-regulation expression of miR-212-3p. ***P < 0.001

### 3.4. PGF was a direct target gene of miR-212-3p

Compared with HC group, both the protein and mRNA expression of PGF in the FGR group were significantly down-regulated (Figure 4(a–b)). In addition, the mRNA expression level and protein expression of PGF were increased When miR-212-3p expression was downregulated (Figure 4(c–d)). And the expression of PGF had negative correlation with miR-212-3p in FGR (Figure 4(e)). Furthermore, PGF could be one of the target genes of miR-212-3p according to the TargetScan database (http://www.targetscan.org/vert_72/) (Figure 4(f)). The results of dual-luciferase reporter assay confirmed that miR-212-3p mimics only inhibited the luciferase activity of PGF-WT, suggesting that miR-212-3p could bind to PGF 3ʹUTR (Figure 4(g)).

**Figure 4.** miR-212-3p can target and regulate PGF

(a) Expression levels of PGF and mRNA in the FGR and HC groups detected by qRT-PCR, *** P < 0.001; (b) PGF expression in the HC and FGR groups detected by Western blot, ***P < 0.001; (c) PGF expression detected by qRT-PCR, ***P < 0.001; (d) PGF expression detected by Western blot, ***P < 0.001; € Negative correlation of miR-212-3p with PGF on the mRNA expression; (f) PGF mRNA and miR-141-3p sequence were schematically depicted; (g) Verification of the target connection between PGF and miR-212-3p detected by Dual-luciferase reporter assay, **P < 0.01.

### 3.5. miR-212-3p downexpressed alleviates si-PGF-induced HTR-8/SVneo functional effects

To determine whether miR-212-3p regulates HTR-8/SVneo cell function by targeting PGF, we performed rescue experiments. As shown in Figure 5(a–c), interference with PGF expression in HTR-8/SVneo cells significantly reduced proliferation, migration and invasion ability and significantly increased apoptosis compared to NC group. However, low expression of miR-212-3p could reverse the functional effects of si-PGF on HTR-8/SVneo cells. These results indicate that miR-212-3p could target PGF to regulate HTR-8/SVneo cell proliferation, migration, invasion and apoptosis in FGR.

**Figure 5.** Reversion of the functional effects of PGF down-regulation on HTR-8/SVneo by down-regulation expression of miR-212-3p

(a) Cell proliferation detected by MTT assay; (b) Apoptosis detected by flow cytometry and quantitative analysis; (c) Cell invasion and migration detected by Transwell assay, ** P < 0.01, ***P < 0.001; ##P < 0.01 and ###P < 0.001.

## 4. Discussion

FGR, being as the main reason of the perinatal morbidity [23], does not have appropriate means for prevention and treatment due to its unclear occurrence and development molecular mechanism. The placenta connects the mother to the fetus and plays a fatal role in the growth of fetal. Many miRNAs have been found to be associated with placental dysfunction. Therefore, we examined miR-212-3p expression levels in placental tissues with FGR as well as normal placental tissues, respectively, and found that expression levels of miR-212-3p were notably higher in placental tissues with FGR. Further interrogating the influence ofmiR-212-3p in FGR, we found the promotion effect of down-regulation expression of miR-212-3p on the invasion, migration and proliferation of HTR-8/SVneo and apoptosis inhibition.

PI3K/AKT signaling pathway is closely related to body life activities and can regulate various life processes such as cell proliferation, protein synthesis and its function, PTEN is inhibited in a variety of tumors, and activated PTEN can inhibit PI3K/AKT activation, which in turn affects a variety of life activities [24,25]. Protein kinase AKT is closely related to cell proliferation, apoptosis, energy metabolism, inflammatory response, immune regulation, and autophagy [26,27], and PI3K, as a phosphatidylinositol kinase, can increase the site phosphorylation level of its downstream important target gene AKT thereby promoting AKT activation [28]. It has been found that PI3K/AKT pathway participates in biological processes including protein synthesis and cell migration in trophoblast cells, indicating that PI3K/AKT pathway has an important role in trophoblast cells [29,30]; By activating the PI3K/AKT pathway, miR-223-3p can significantly enhance the invasion, migration and proliferation of trophoblast cells, indicating that miRNA is of a great importance in trophoblast cell activity through the regulation of PI3K/AKT pathway [31]. Down-regulation expression of miR-212-3p notably raised the expression levels of p-AKT and p-PI3K in cells which in turn activated the signaling pathway of PI3K/AKT. Zhang et al. [32] similarly found that miR-362-5p promotes HTR-8/SVneo cell proliferation and inhibits apoptosis by targeting glutathione disulfide reductase (GSR) and activating the PI3K/AKT pathway. These studies suggest that miRNAs can exert effects on trophoblast cell function by regulating the PI3K/AKT signaling pathway. We have come to the same conclusion. In the present study, we found that downregulation of miR-212-3p expression significantly increased the protein phosphorylation expression of PI3K and AKT in HTR-8/SVneo cells, which in turn activated the PI3K/AKT signaling pathway. It was revealed that miR-212-3p could regulate the biological functions of HTR-8/SVneo cells through PI3K/AKT signaling pathway.

Further, according to the previous bioinformatics experiments, it was found that PGF was the target gene of miR-212-3p. PGF, which belongs to the vascular endothelial growth factor family, is a proangiogenic protein [33,34]. Its expression is closely related to the interaction between vascular cells, trophoblasts and endothelial cells [35]. Some studies have found that PGF levels are significantly lower in growth-restricted placental tissue compared with normally growing placental tissue [36]. In addition, PGF induces malignant biological behaviors such as trophoblast invasion as well as phosphorylation reactions [37]. Tao et al. [38] revealed that miR-124-3p inhibited HTR-8/SVneo cells invasion and migration but increased cell pyroptosis via targeting PGF. In this study, PGF was found to be significantly decreased in FGR, which corresponds with previous researches [36]. Besides, we also confirmed that in FGR tissues, PGF expression was negatively correlation with miR-212-3p expression. To further confirm the relationship, luciferase activity assay confirmed the presence of targeting between PGF and miR-212-3p. PGF knockdown reduced HTR-8/SVneo cells proliferation, migration and invasion ability, and increased cell apoptosis. More importantly, we also found the reversion effect of si-PGF on HTR-8/SVneo by down-regulation expression of miR-212-3p. suggesting that miR-212-3p promoted apoptosis but decreased invasion and migration of HTR-8/SVneo cells via targeting PGF.

## 5. Conclusion

We demonstrated that miR-212-3p is upregulated in FGR and targets PGF, inhibiting trophoblast cell proliferation, migration and invasion but promoting apoptosis by regulating the activity of PI3K/AKT signaling pathway. This provides a new molecular marker for the diagnosis and treatment of FGR.

## Highlight

1. High expression of miR-212-3p and low expression of PGF in placental tissue with fetal growth restriction.
2. Low expression of miR-212-3p promotes proliferation, invasion and migration of HTR-8/SVneo cells and inhibits apoptosis.
3. miR-212-3p targets PGF.
4. miR-212-3p downregulation activates the PI3K/AKT signaling pathway.
